# Intelligent Simulation of Children's Psychological Path Selection Based on Chaotic Neural Network Algorithm

**DOI:** 10.1155/2021/5321153

**Published:** 2021-09-29

**Authors:** Yue Wang

**Affiliations:** School of Education, Zhongyuan Institute of Science and Technology, Zhengzhou, Henan Province 450046, China

## Abstract

In recent years, there are many problems in the study of intelligent simulation of children's psychological path selection, among which the main problem is to ignore the factors of children's psychological path selection. Based on this, this paper studies the application of chaotic neural network algorithm in children's mental path selection. First, an intelligent simulation model for children's mental path selection based on chaotic neural network algorithm is established; second, it will combine the network based on different types of visual analysis strategies. The model is used to analyze the influencing factors of children in different regions in the choice of psychological paths. Finally, experiments are designed to verify the actual application effect of the simulation model. The results show that compared with the current mainstream intelligent simulation methods with iterative loop algorithms as the core, it adopts the intelligent simulation model based on the chaotic neural network algorithm has a good classification effect. It can effectively select the optimal psychological path according to the differences in children's personality and can adaptively classify children in different regions, and the experimental results are accurate. Compared with the traditional method, it is improved by at least 37%.

## 1. Introduction

The intelligent development of children's psychological path selection is based on caring for the healthy growth of children, which is not a new word [1]. Although it has been developed for many years, it has not formed a fixed standard and model [2]. At present, there are many research methods for children's psychological path selection, but generally through the collection of children's scattered behavior and personality information and the data set analysis and deep learning to achieve the intelligent simulation of children's psychology [3]. The core content of the simulation of children's psychological path selection lies in the accurate analysis of various factors that affect children's choice, then, according to the corresponding conditions, reasonable distribution of the proportion of each factor, and finally get the optimal children's psychological path selection [4].

The innovation of this paper lies in the chaotic neural network algorithm and how to establish the relevant model based on this algorithm. The simulation model established by the algorithm can realize the automatic classification of children in different regions and different family conditions in the same region and design different screening models according to this, which greatly increases the accuracy of the model.

This paper studies the application of chaotic neural network algorithm in the intelligent simulation of children's psychological path selection, which is mainly divided into four sections. In Section 2, the related work in the field is introduced. In Section 3, an intelligent simulation algorithm model based on a chaotic neural network algorithm is constructed. The model can automatically classify children's psychology according to different cultural characteristics of different regions and economic characteristics of different families in the same region. In Section 4, the application of the intelligent simulation child selection model in intelligent recognition and classification of children with different conditions is tested. The experimental results and errors are analyzed, and the conclusion is drawn; compared with the traditional model, the proposed model based on a chaotic neural network algorithm has higher accuracy and recognition speed. In Section 5, this paper is concluded, and some suggestions are listed.

## 2. Related Work

In recent years, people's research on children's psychological path selection has made great progress,. However, the current mainstream psychological path selection algorithm is complex and the model speed is slow, resulting in the final model not achieving the desired effect of researchers. When establishing the intelligent selection model, Nunes et al. relied on the universal algorithm, which has the problem of nonpertinence, that is, they do not consider the different psychological characteristics of children in different regions, so the algorithm often does not have pertinence, which leads to the model can't match the psychological characteristics of children in different regions [5]. Mahmud et al. found that this kind of intelligent algorithm belongs to a high energy consumption algorithm, which has great difficulty in data stability [6]. Gorban et al. used the traditional iterative algorithm in model design, which did not fully consider the constraints, resulting in the established model that does not meet the requirements in terms of speed or accuracy [7]. In addition, according to Goldberg et al. in the study of children's psychology, there are many unreasonable places, such as a large number of copying city psychological models and even some adult psychological models, which leads to the establishment of the model not only does not conform to the psychological characteristics of children [8]. Nadeem et al. believe that different types of factors will seriously interfere with other scholars' research on intelligent simulation of children's psychological path selection [9]. In order to improve the operation speed of the model, Zeman et al. have established a basic emotional model, but the model only designs some simple psychological choice paths, resulting in the model that does not conform to the real psychological characteristics of children [10]. Halverson et al. have designed models based on multiple environment algorithm to classify children in different regions [11]. Spratt et al. found that children with different family conditions in the same area were not distinguished, which affected the accuracy of the results of the intelligent selection algorithm [12].

In summary, it can be seen that the current intelligent simulation children's psychological path choice model generally has problems such as poor classification effect, low classification accuracy, poor stability, and low data utilization [13, 14]. On the other hand, the current mainstream intelligent simulation methods with iterative loop algorithms as the core are processed. In the existing children's mental intelligence selection models, most of them are based on the results of multidimensional linear analysis strategies. Therefore, most of the model algorithms are too complicated. The model calculation speed is slow, and the energy consumption is huge, which cannot meet the needs of fast and low energy consumption [15]. And in the process of building models in the past, due to mistakes borrowing from other mental models, more erroneous data were obtained [16].

## 3. Methodology

### 3.1. Application of Chaotic Neural Network Algorithm in Intelligent Simulation of Children's Psychological Path Selection

Algorithm expression ability is an important skill that researchers cannot ignore, and models designed under the same algorithm will have different forms of expression [17]. The expression of chaotic neural network algorithm is to show the constructed model with the help of various media to convey the design intention and model structure [18]. From design conception to model construction, we need to combine design thinking and algorithm thinking closely. Whether it is the method of children's psychological path selection or the performance of different dimensions of computer data types, it is an important means of performance model [19]. At present, the expression forms of models constructed by chaotic neural network algorithm begin to show diversified development, among which computer animation, computer frame, and hand-drawn effect picture are the most common three types of model expressions [20].

Chaotic neural network algorithm is a kind of data solution promoted in recent years. Compared with other common algorithms, this method pays more attention to data analysis conception and data processing innovation [21]. With the development of computer digital technology, the idea of chaotic neural network algorithm has been paid more attention, and it has become an indispensable way of expression in the intelligent simulation of children's psychological path selection [22]. In the overall design scheme of the model, researchers need to carry out computer data simulation creation to show the effect of selection analysis [23]. Computer data analysis technology has good color effect, three-dimensional space effect, and stronger performance ability and can simulate the real selection process [24]. This performance method is convenient and fast, and it does not require high drawing technology for researchers. It is convenient for researchers to quickly correct the selection results manually. This is because the core technology of the chaotic neural network algorithm is the underlying technology of the neural network algorithm.

### 3.2. Modelling Process of Chaotic Neural Network Algorithm

In this study, chaotic neural network algorithm from the perspective of children's psychological construction summarizes children's psychological characteristics in detail, so as to ensure that children's normal healthy thinking can be inherited and selected. In the algorithm design, we need to go deep into the neural network, understand children's way of thinking, and analyze the establishment process of the neural network. On the other hand, we also need to integrate the regional characteristics into the algorithm to fully reflect the rationality of children's psychological path selection [25]. On this basis, the research of the intelligent algorithm, on the basis of the establishment of chaotic neural network style, fully reflects the normal psychology of children. In the design process, we should make full use of advanced algorithm technology, constantly improve the reliability of deep learning, and retain the integrity of the intelligent algorithm to ensure its advanced nature. The classification principle is an important principle in the design of children's psychological path selection based on chaotic neural network. According to different children's psychological conditions and external conditions, the correct results for the children are formulated. Children in different regions have different psychological characteristics, external conditions, and psychological styles. Therefore, we need to follow the principle of classification and fully combine the factors of different cultures and economic levels. For example, the geographical and economic factors should be fully considered in the design of children's psychological path selection in mountainous areas, which will account for a higher proportion of the influencing factors. In the process of establishing the basic algorithm module of neural network, the regional condition is an important condition that can be used, and it is also an important way to maintain the local characteristics. Therefore, in the design, the characteristics of the original intelligent classification should be fully guaranteed, and valuable psychology should be preserved. The data analysis process is shown in Figure 1.

The chaotic neural network algorithm proposed in this research is to directly give each neuron the chaotic properties, that is, changing a chaotic iterative function is equivalent to finding a “new” neural network. The chaotic nature is achieved through explicit or implicit iteration. Through chaotic iteration, the internal state variables of the neuron at a continuous-discrete time *t*, *t *+* *1, *t *+* *2,… can be associated, and the weighted sum of all other neuron outputs can be processed as input. The design of children's psychological path selection based on chaotic neural network should fully follow the concept of intelligent design, make full use of scientific resources and artificial algorithms according to the biological principles of nature, and realize children's psychological intelligent selection. In terms of psychological path and intelligence, the construction of a chaotic neural network has great development potential. In the design of children's psychological path selection, we should make full use of the existing algorithm resources and model resources. Neural network algorithm resource is abundant; we can consider the decentralized learning methods together, improve the intelligent level of the model, and improve the computational efficiency. In the design of intelligent path selection, we need to keep the old algorithm with research value. When designing the new algorithm, we should make full use of the link algorithm to connect, ensure the overall harmony of each part of the neural network, and avoid serious old differentiation. We encourage the chaotic neural network to implement an intelligent selection system in the new algorithm and adjust the selection mode while obtaining the correct results, so as to improve the quality of the model results.

There are great differences in culture among different places. Each place has its own regional culture. The existing children's psychological path intelligent selection model often uses the common urban psychology, most of the common algorithms, do not reflect the regional culture and environmental characteristics, ignore the cultural connotation, and destroy the correctness of the results, resulting in the lack of regional characteristics and cultural integrity. In the past, the common models did not show differences from other regional cultures and lack of regional cultural differences. The research of intelligent simulation children's psychological path selection should be people-oriented, fully consider the living habits of children in different regions, and build a psychological path model suitable for children in different regions. All kinds of algorithm design should be able to meet all kinds of functional requirements. From the perspective of deep learning, the needs of learning depth should be fully considered. In the process of selecting a deep learning training sample set, we should fully combine the psychological needs of children in different environments and adopt an independent design method. In the process of neural network design, we can add the necessary lateral algorithm branches. The multiple iterative algorithm is the way often used before. Now we can still use this way to increase the lateral branches of chaotic neural network and then expand the application scope and accuracy of the model.

### 3.3. The Establishment Process of Children's Mental Path Selection Intelligent Simulation Model Based on Chaotic Neural Network Algorithm

The children's mental path selection design effect image to be classified is analyzed, and the most visual feature image is taken as the training sample. The reasonable algorithm is used to extract, and multiple feature values are obtained. Then, the eigenvalues are normalized, the classification mechanism is selected, the training set is used for training, and the classification results are obtained. The data training and classification process based on a chaotic neural network is shown in Figure 2.

In addition, the algorithm proposed in this research can directly transform the classic neural network, using the existing learning algorithm to make the classic neural network (such as the network with hidden layers) learn the chaotic attractor (such as the use of Ikeda chaotic attractor) to allow the network to simulate the orbit of the chaotic attractor to a certain extent and then introduce methods such as delay feedback control to enable the network to have chaotic behavior. The input is the children's psychological test data, and the output is the children's psychological path test analysis report data group. The differences in children's mental path selection design renderings are mainly reflected in the color, texture, and other aspects of mental health. Color is an important visual element, and extraction is relatively simple. Color histogram is one of the typical color features, which reflects the intensity of color. The color histogram *Q* can be expressed as follows:

(1) $$\begin{array}{c} Q=\sum_{i=1}^{n}b_{i}^{2}!, \end{array}$$

where *b* is the intensity, and the color histogram is an important color feature used in many algorithms. By analyzing the features of each image, generally speaking, the number of colors contained in hand-drawn and white images is small, so it is necessary to extract quantitative features from the sample images. The simulation results are shown in Figure 3.

As can be seen from Figure 3, with the change of data types, the differences of quantitative features are also different, but the differences are obvious. This is because, for color images, it is necessary to extract them in a specific space. Assuming that *g* and *v* are the reference color points in RGB space, *r* and *W* are the color points in HSV space; the space transformation should meet the following requirements:

(2) $$\begin{array}{c} s=\sqrt{v}\frac{\sum_{i=1}^{n}b_{i}^{2}!}{r!\left(g-r\right)!}. \end{array}$$

Color histogram of HSV space is used to reflect color features, and HVS space is quantized. In the experiment, the hue *H* is divided into 8 parts, and the saturation and brightness are divided into 3 parts. HSV quantizer was used for processing. Each color component composes a feature vector.

(3) $$\begin{array}{c} L=\underset{s⟶\infty }{\lim}\sqrt{H^{2}+V^{2}}+3S. \end{array}$$

In the formula, the range of *L* is 0 ∼ 71, and the color pixel array of different color levels is composed of 72 color histograms, reflecting the statistical characteristics of the image.

The computer rendering uses a more realistic texture to show the design, so it has higher saturation. Combined with the previous research on the intelligent simulation of children's psychological path selection, RGB color space is converted to HSV color space. There are *L* saturation in the range of 0 ∼ 1, and the histogram is a discrete function

(4) $$\begin{array}{c} f\left(S_{k}\right)=\underset{k⟶\infty }{\lim}n_{k}, \end{array}$$

where *S*_*k*_ is saturation and *n*_*k*_ is the number of pixels in the image. After the color conversion space is completed, the data is normalized:

(5) $$\begin{array}{c} P\left(S_{k}\right)=\frac{\sqrt{h{\left(S_{k}\right)}^{2}+n^{2}}}{n}, \end{array}$$

where *n* is determined according to the basic knowledge of probability theory, the frequency of *P*(*S*_*k*_) reaction saturation. The optimal eigenvalue is selected to analyze the rendering image as follows:

(6) $$\begin{array}{c} R_{L-1}=\frac{\sum PDS_{L}}{P\left(\sqrt{2}S_{1}\right)}. \end{array}$$

Assuming that the separable measure of *R*_*L*−1_ is represented by *S*_*L*_, the larger the *S*_*L*_ is, the better the separability of samples is. A feature is proposed from *R*_*L*−1_, which can retain the maximum eigenvalue. In this study, *P*(*S*_*L*_) is set to 0.9, and the simulation results are shown in Figure 4.

As can be seen from Figure 4, with the change of data type, although the curve change trend is similar, the numerical results show different differences. This is because in the simulation process, the image can be divided into nonlinear separable and linear separable. For a consistent linear separable data set, the sample feature vector belongs to *g*(*x*), and *x* is used to represent the class label, which contains two types of samples. The linear discriminant function in d-space can be expressed as follows:

(7) $$\begin{array}{c} g\left(x\right)=w\sqrt{x}+bx. \end{array}$$

The classification line is required to classify all samples accurately; the following conditions should be met:

(8) $$\begin{array}{c} \frac{y_{i}\left[\left(wx_{i}\right)+n\right]}{\sqrt[{3}]{w}}\geq 0. \end{array}$$

This can ensure that the smallest classification surface is the best surface. The training sample points on the chaotic training set are the optimal vectors selected by the neural network; the optimal neural network function is expressed as follows:

(9) $$\begin{array}{c} f\left(x\right)=\mathrm{sgn}\left\{\sum_{i=1}^{n}a_{i}y_{i}\left(x_{i}\times x\right)+b^{*}\right\}, \end{array}$$

where sgn is the sign function, *a*_*i*_ is the optimal solution, and *b* is the classification threshold.

If the training samples are not linear separable samples, the above methods cannot be adopted, so it is necessary to add relaxation terms and constraints as follows:

(10) $$\begin{array}{c} \frac{y_{i}\left[Dw\times x_{i}+b\right]-1}{\sqrt{\zeta_{i}}}>0. \end{array}$$

Under this condition, the minimum value *ϕ*(*w*, *ζ*) of *ϕ* is calculated as follows:

(11) $$\begin{array}{c} \phi \left(w,\zeta \right)={\left\|w^{2}\right\|}^{3}+\frac{2}{3}C\left(\sum_{i=1}^{n}\zeta_{i}\right), \end{array}$$

where *C* is the additional error cost coefficient, which reflects the penalty degree of misclassification samples.

In the construction of the optimal interface, the original space is realized in the high-dimensional space. After the optimal interface is determined, the given training samples belonging to two categories can be separated, and the chaotic vector machine learning algorithm can be constructed between the chaotic vector and the output vector. At present, there are four kinds of kernel functions, which can be selected reasonably according to the actual situation. After introducing the kernel function, the decision classification function is transformed into

(12) $$\begin{array}{c} f\left(x\right)=\mathrm{sgn}\left\{w^{*}\times \sin^{-1}\;x+b^{*}\right\}. \end{array}$$

In this paper, we need to introduce a binary-tree-based chaotic vector machine classifier. The specific process is to divide all categories into two categories according to the different features and divide the image into two categories and each subclass into two subclasses, so as to cycle until the optimal result is obtained.

The training classification area of the chaotic neural network generates a training sample set according to the feature vectors of children's mental path selection design effect picture. Each sample file contains all the feature vectors and symbols and then determines the classification model. After normalization, the feature data are sent to the chaotic neural network for data preparation, and the kernel function and other parameters need to be determined. Generally, a radial basis kernel function is preferred as follows:

(13) $$\begin{array}{c} G\left(x_{j},x_{i}\right)=\underset{\delta x⟶0}{\lim}\left\{\frac{\sqrt{\left|x_{i}-x_{j}\right|}}{\delta^{2}}\right\}. \end{array}$$

After determining the kernel function, we need to determine the parameters of the kernel function itself and the error cost parameters. The cross-validation method is used to determine the optimal parameters, and the simulation results are shown in Figure 5.

As can be seen from Figure 5, with the increase in the number of samples, the simulation results show different changes. This is because after the sample features are divided into a training set and a verification set, the classification accuracy calculated will also be different. Therefore, this paper selects the *K*-fold cross-validation method; for the sample data set, it is divided into *k* nonintersecting subsets and then verified, using different subsets as the test set, and the rest as the training set.

## 4. Result Analysis and Discussion

### 4.1. Experimental Design of Children's Psychological Path Selection Model Based on Chaotic Neural Network Algorithm

In the process of experiment, the intelligent simulation model designed by chaotic neural network algorithm should have the function of classifying different children's personality characteristics. In the process of building the main body model, the design options need to meet the needs of personality and hobbies. At the same time, the model also needs to set up the necessary neural network branches and horizontal and vertical iterative algorithm branches to increase the characteristics of different places [26–30]. After determining the best parameters, the images of the intelligent simulation model are automatically classified, and a total of 400 samples are collected, covering computer animation, black and white performance, computer performance, and so on. The design pictures are selected as the training image set, and different forms of artistic expression are marked. Combined with the binary tree, the typical eigenvalues of the training samples under four chaotic vector machines are obtained, and the training sample files are generated. The remaining images are classified as test images. By reading the test image classification results and outputting them to the interface, the classification accuracy is obtained. In the process of building the branch model, we should pay attention to the function space of each part of the model, separate the external conditions from the internal conditions, and pay attention to the different functions produced by different options and different environments.  Figure 6 is the preliminary experimental results of the branch model of chaotic neural network algorithm.

In the four sets of data in Figure 6, the three different methods have different branch accuracy indicators for the processing results of the data, and the branching degree of the results obtained under the processing of the chaotic neural network algorithm is the lowest (the lower the value represents its stability, the better the result), and it also best meets the experimental requirements. It can be known that the processing result of the chaotic neural network algorithm proposed in this research is the best. As can be seen from Figure 6, in the internal space design, combined with the actual situation of children, we can adopt both compact design and multifunctional design to minimize the instability of chaotic neural network. There is the problem of error storage in the model space of children's neural network, so we need to set up the necessary additional algorithm storage space. We can consider the method of developing the algorithm branch of a chaotic neural network to solve these problems, which is mainly used to store the judgment conditions. Therefore, in the process of the experiment, the internal algorithm design adopts the deep learning mode of classification to avoid blindly following the trend.

### 4.2. Experimental Results and Analysis

The evaluation index proposed in this research is frequency statistics [31–35]. The evaluation process is that in the iterative process, if the Hamming distance between the output of the network and a memory vector is 0 (or close to 0) frequently, it can be considered that the memory vector is successfully identified. If the Hamming distance between the output of the network and multiple memory vectors is 0, it is considered that the memory vector with the most Hamming distance of 0 is identified. The intelligent algorithm is used to analyze the experimental results and extract the information. Because the parameters, sample number, and kernel function are different, the normalization methods used are very different, so the classification results are also different. The binary tree chaotic vector machine classifier algorithm is taken as an example to determine the reasonable parameters. In the parameter determination, the selection is made from the angle of classification accuracy to ensure the highest classification accuracy. In classification, data normalization plays an important role, and it also affects the overall success or failure. In the study, it is assumed that the number of training samples is 50, the number of test samples is 40, and the penalty factor is set to 70. The experimental results are shown in Figure 7.

As can be seen from Figure 7, different neural network optimization methods can be preprocessed to obtain the reference value of the classification accuracy index (the limit is set to 0.54). Through the experimental analysis, we can see that the normalization method can significantly improve the accuracy. If the classifiers are the same in the same data set, but the results are different, it is considered that the data is not normalized. From the data in the table, we can see that the classification accuracy is the highest after normalization in [−1, 1].

Kernel function has strong generalization ability, as long as it can satisfy Mercer's function, it can be used as a kernel function. However, the classification performance of different kernel functions is different. When selecting the kernel function, other parameters are selected, the training sample size is set to 50, and the normalization processing is carried out in [−1, 1]. The classification accuracy of the two models can be compared and analyzed.  Figure 8 is the classification accuracy measurement results.

It can be seen from Figure 8 that among the three methods, compared with the other two methods, the mental path selection model error index obtained by the chaotic neural network algorithm is the lowest (regardless of the change in the number of analyses) and shows a gradual decrease. Therefore, the model accuracy rate is the highest in the chaotic neural network optimization method. It can be seen from Figure 8 that the accuracy of the model is the highest when the radial z-basis function is the chaotic neural network optimization method. This is because, in the selection of various parameters of the chaotic vector machine, it is generally determined by different kernel functions and corresponding parameters. Take *K*_*A*_ as an example, the kernel function is randomly selected as the parameter value, the *C* value is 2, and the random parameter *δ* is 2, The accuracy is 90% when the random parameter *δ* value is 1; *C* = 10, and the random parameter *δ* is 1. The accuracy was 82.5%; *C* = 20, and the random parameter is 10. The accuracy was 77.5%; *C* = 50, the random parameter *δ* is 50, and the accuracy was 67.5%; *C* = 70. The accuracy is 90% when the random parameter *δ* is 5.

It can be seen from the experimental data that the classification performance is different with different parameters. It is found that the smaller the C is, the better the sample number is, the larger the value *δ* is, the larger the chaotic neural network tends to be linear. Therefore, the CV can be used to find the best parameter.  Figure 9 shows the curvature change of accuracy.

It can be seen from Figure 9 that as the number of iterations increases, the optimal fitness gradually increases. Among the three methods, the accuracy of the mental path selection model obtained by the chaotic neural network method is much higher than that obtained by other methods. As a result, the amount of data required when the maximum value is reached for the first time is significantly smaller than that of the other two methods. This is because the number of samples is different, which will also affect the accuracy of automatic classification. According to the number of samples, it can be divided into large samples and small samples. The sum of all possible observation results is the population. In this paper, when the number of samples is more than 30, the sample is large; otherwise, it is small. Taking the experimental data in this study as an example, 120 children's mental path selection design pictures are selected to form a sample library, including digital performance and hand-painted pictures. Forty samples are selected for each category as the test set, and the remaining samples are used as the training set to test the classification accuracy. Therefore, there are many parameters that affect the accuracy; the sample size will affect the accuracy of the experimental results; and the change trend of the two is basically consistent.

## 5. Conclusion

In recent years, there are many problems in the study of intelligent simulation of children's psychological path selection, among which the main problem is to ignore the factors of children's psychological path selection. Based on this, this paper studies the application of chaotic neural network algorithm in children's mental path selection. First, an intelligent simulation model for children's mental path selection based on chaotic neural network algorithm is established, combined with network models based on different types of visual analysis strategies for analysis influencing factors of children in different regions in the choice of psychological path, and finally designed experiments to verify the actual application effect of the simulation model. The results show that compared with the current mainstream intelligent simulation methods with iterative loop algorithms as the core, chaotic neural networks are used. The intelligent simulation model of the algorithm has a good classification effect, can effectively select the optimal psychological path according to the differences of children's personalities, and can be adaptively classified for children in different regions, and its experimental results are more accurate than traditional methods at least 37%. But the shortcoming of this article is that this research only analyses from the perspective of automatic classification of children's mental design effect maps, and other aspects need to be discussed and analyzed in depth.

## Figures and Tables

**Figure 1:** Chaotic neural network data analysis process.

**Figure 2:** Data training and classification process based on chaotic neural network.

**Figure 3:** Simulation analysis results of different types of children's mental health data.

**Figure 4:** Simulation analysis of children's mental path selections under different degrees of completion.

**Figure 5:** Cross-validation results under different data analysis simulation completion levels.

**Figure 6:** Preliminary experimental results of chaotic neural network algorithm model.

**Figure 7:** Experimental analysis results.

**Figure 8:** The algorithm obtains the uncertainty of choice.

**Figure 9:** Accuracy changes under different iteration times.

## Data Availability

The data used to support the findings of this study are available from the author upon request.
